This article has been retracted.

# Evaluation of the Effectiveness of a Combination of Chinese Herbal Fumigation Sitz-Bath and Red Ointment in Managing Postoperative Wound Healing and Pain Control in Anal Fistula Patients

**DOI:** 10.1155/2022/1905279

**Published:** 2022-09-15

**Authors:** Li He, ZhiLing Yang, Jin Xu, QingMing Wang

**Affiliations:** ^1^Department of Traditional Chinese Medicine, Shanghai Tenth People's Hospital, Shanghai 200072, China; ^2^Department of Anorectal Diseases, Shanghai Baoshan Integrated Traditional Chinese and Western Medicine Hospital, Shanghai 201900, China; ^3^Department of Anorectal Diseases, Shuguang Hospital Affiliated to Shanghai University of Traditional Chinese Medicine, Shanghai 201203, China

## Abstract

**Objective:**

To explore the efficacy of Chinese herbal fumigation and sitz-bath combined with red ointment in the treatment of postoperative wound healing and pain control in anal fistula patients.

**Methods:**

A total of 118 anal fistula patients were selected as the study population, randomly divided into two groups, i.e., the research group (*n* = 60) and the control group (*n* = 60). The control group was treated with red ointment therapy for postoperative wound healing and pain while the research group was treated with a combination of ointment and traditional Chinese medicine fumigation sitz-bath, Postoperative wound healing, pain control, and safety evaluation were compared between the two groups. Results. The total effective rate in the research group was 96.67%, which was significantly higher than that in the control group (93.10%), and the difference was statistically significant (*P* < 0.05). The VAS scores and postoperative wound healing times in the research group were significantly lower than those in the control group. The difference was statistically significant (*P* < 0.05). A day after postoperative treatment, there was no significant difference (*P* > 0.05) in TNF-*α* and IL-6 levels between the two study groups; however, from day 3 to day 14 the levels were statistically different. TNF-*α* and IL-6 levels in research group were significantly lower than those in the control group. The difference was statistically significant (*P* < 0.05). The incidence of postoperative complications in the research group at 6.67% was statistically significant (*P* < 0.05), significantly lower than 13.79% in the control group. Conclusion. Postoperative intervention with Chinese herbal fumigation and sitz-bath combined with red ointment can effectively reduce the wound healing duration and lower the degree of pain experienced by anal fistula patients, thereby improving their quality of life.

## 1. Introduction

In medical terms, an abnormal opening which leads to the interaction of two or more epithelial surfaces is termed a fistula [1]. Anal fistula is a disease characterised by the interaction of the anorectal canal and the perianal skin which is lined by granulation tissue [2]. Anal fistula occurs at any age; however, peak incidence has been reported in the 20–40-year age group [3]. The incidence of anal fistula is 1,228 in every 100,000 per year, with a higher male incidence compared to that in females [4]. Research studies have indicated that the higher incidence in men can be attributed partially to the greater abundance of anal glands compared to those in females [5].

Anal fistula can be caused by complications of serious bowel diseases such as Crohn's disease [1], tuberculosis [4], infection of anal glands [6], ulcerative colitis [7], and chronic inflammation [8], among other factors. The clinical symptoms of the disease include the rupture of perianal abscess, infection, and pus discharge which all negatively affect the quality of life of patients [9].

At present, an anal fistula cannot heal naturally without any intervention [10]. Surgery is the main treatment for anal fistula [4, 11]. Although surgery is the most effective treatment method to date, the particularity of the anatomical structure presents challenges during and after anal fistula surgery. The majority of postoperative wounds are open wounds which are susceptible to bacterial infections, extremely vulnerable to inflammatory stimulation, and lead to increased peripheral inflammatory exudate. Moreover, the anal region is extremely rich in neurovessels which are highly sensitive to pain, making defecation result in unbearable pain. This continued strain on the affected region causes wound edge fibrosis, anal sphincter spasm, and affects wound healing, creating a vicious circle [12].

Ameliorating the healing quality after anal fistula surgery is, therefore, an important research aspect in anorectal surgery studies. In traditional Chinese medicine, it is believed that the wound healing after anal fistula surgery is difficult because the original surface skin and muscle are damaged. The lesion is removed by surgery, resulting in the local damp-heat pathogens not being exhausted. The wound surface is in a pathological state of stasis, dampness, and heat after surgery. Therefore, the main treatment principles for wound healing after anal fistula surgery should be the removal of rot and muscle, clearing away heat and dampness, promoting blood circulation, and removing blood stasis [13].

Red ointment has been successfully used in the postoperative treatment of anal fistula. The main components in red ointment are Jiu and Dongdan, with the former responsible for clearing heat and muscle, while the latter detoxifies and dispels decay. The traditional Chinese medicine, fumigating and washing sitz-bath is an important method of external wound treatment. It uses the transpiration of medicine [14] to burn the affected area and relies on the action of medicine force and heat to directly contact the diseased area. The medicine force can reach the diseased area to remove pathogens, unblock blood vessels, and reconcile the qi [15].

### 1.1. Related Studies

Previous scholars have used iodophor, infrared radiation, potassium permanganate, and other methods for treatment of anal fistula, but the effect is not ideal [16]. Studies by [17] utilizing the Chinese herbal fumigant with lotion for curing postoperative wounds in anal fistula with results showing great efficacy. Zhang et al. [14] showed that Chinese medicine helps patients recover faster and has fewer side effects than Western medicines.

Due to the flexibility inherent in traditional Chinese medicine [18], there are endless possibilities for its application in treating anal fistula. However, there is no study at home or abroad that explores the effect of traditional Chinese medicine fumigating and bathing combined with red ointment on postoperative wound healing of anal fistula patients. Therefore, this study retrospectively analyzed the clinical data of 118 patients with anal fistula who received surgical treatment in our hospital so as to provide a new scheme for the recovery of patients with anal fistula.

## 2. Material and Methods

### 2.1. General Material

Research subjects were selected from patients with anal fistula who underwent surgical treatment in our hospital from March 2019 to October 2021. A total of 118 patients aged between 21 and 58 years were selected and divided into 2 groups according to the treatment methods adopted. The control group had 58 patients who were treated with conventional treatment using red ointment, while 60 patients in the research group were treated with a combination of traditional Chinese medicine fumigation and sitz-bath with red ointment. Ethical approval for undertaking this study was acquired from the departmental ethics committee.

### 2.2. Criteria for Inclusion and Exclusion

Inclusion criteria:(1) Patients meeting the diagnostic criteria in the Consensus of Chinese Experts on Anal Fistula Diagnosis and Treatment (2020) [19]; (2) Age ≥20 years; (3) patients who met the indications for anal fistula surgery and underwent one-stage resection; and (4) patients with complete clinical data.

Exclusion criteria: (1) Patients with other anorectal diseases; (2) patients with previous anorectal surgery; (3) patients with cognitive impairment who did not cooperate with follow-up; and (4) patients with malignant tumors or organ dysfunction.

### 2.3. Research Methods

Patients in the control group were treated with red ointment constituted by 30 g of Jiu Yi Dan and 4.5 g of lead Dan with an appropriate amount of vaseline ointment on a dry gauze. The red ointment gauze was evenly applied on the wound surface twice a day after high-pressure steam disinfection.

The research group was treated with traditional Chinese medicine fumigating and washing sitz-bath whereby heat-clearing and pain-relieving soup and fumigating and washing sitz-bath were used on the wound before treating with red ointment. The red ointment treatment protocol was similar to the one used in the control group. The Chinese medicine soup drug was composed of 20 g of raw rhubarb, 20 g of Smilax glabrata, 15 g of schizotuina, 60 g of Houttuynia cordata, and 20 g of Rhizop.

### 2.4. Observational Measurements

1. Evaluation of curative effect: A cure is confirmed by the disappearance of clinical symptoms and signs. The wound healed well and the pus-rot tissue fell off; the obvious effect was that the clinical symptoms and signs were significantly ameliorated compared with those before treatment; the wound area was reduced by ≥ 75%, the pus-rot tissue basically fell off, and the pain was relieved; the effective effect was that the clinical symptoms and signs were significantly ameliorated compared with those before treatment, and the 75%> wound area was reduced by ≥ 30%, and the pain was tolerable. Other symptoms did not ameliorate.
2. Pain evaluation, using pain visual analog scale (visual analogue scoring of pain, VAS) [20] to evaluate the degree of pain in the two groups of patients, 10 points for severe pain, 0 points for pain, 3 days after surgery, 7 days after surgery, and 14 days after surgery.
3. Wound granulation evaluation, referring to the ulcer scoring principle in the relevant literature [21], even if granulation tissue grows vigorously, the wound bulge is 0 points, the granulation tissue grows vigorously, the wound flat is 1 point, the granulation tissue grows slowly, and the wound depression is 2 points. The granulation growth was evaluated 3 days, 7 days, and 14 days after operation.
4. Comparison of wound healing time was noted, recording the number of days from the date of operation to complete wound healing.
5. Evaluation of wound exudate and edema, referring to the evaluation criteria of surface exudate and edema in the relevant literature [22]. The score range is 0–3. The higher the score, the better the recovery. Wound exudates and edema were evaluated 3 days, 7 days, and 14 days after surgery.
6. Assessment of inflammatory factors. Fasting elbow venous blood of 5 ml was collected 3 days, 7 days, and 14 days after operation, centrifuged for 15 min at 3000r/min. The supernatant was taken and the levels of interleukin-6 (Interleukin-6, IL-6) and tumor necrosis factor-*α* (TNF-*α*) were measured by enzyme-linked immunosorbent assay.
7. A safety evaluation and comparison of the incidence of adverse complications during treatment between the two groups was conducted.

### 2.5. Statistical Methods

SPSS version 20.0 was applied for data processing while statistical graphs were developed using GraphPad Prism version 9. The comparison of count data between the two groups was expressed as (*n* or %) using the chi-square test. The comparison of count data between the two groups was expressed as standard deviation ± mean (*x* ± *s*), using the *t*-test. The difference was statistically significant if *P* < 0.05.

## 3. Results

### 3.1. Comparison of Baseline Information between the Two Groups

There was no significant difference between the two groups in age, course of disease, and sex (*P* > 0.05), as shown in Table 1.

### 3.2. Comparison of Efficacy between the Two Groups

The total effective rate of the research group was 96.67% which was significantly higher than that of the control group (*P* <93.10%), and the difference was statistically significant (*P* < 0.05), as displayed in Table 2.

### 3.3. Comparison of Pain Scores between the Two Groups

The VAS scores of the two groups improved significantly after operation and gradually improved with the increase of time. The VAS scores of the research group were significantly lower than those of the control group between 3 days and 14 days after operation, and the difference was statistically significant (*P* < 0.05), as manifested in Table 3 and Figure 1.

### 3.4. Comparison of Wound Healing Time between the Two Groups

The wound healing time of the research group was significantly lower than that of the control group (*P* < 0.05), as shown in Table 4 and Figure 2.

### 3.5. Comparison of the Growth of Granulation in Wounds between Two Groups

The granulation growth score of the two groups alleviated significantly after operation, and alleviated gradually with the increase of time. The granulation growth score of the study group was significantly lower than that of the control group between 3 days and 14 days after operation, and the difference was statistically significant (*P* < 0.05), as shown in Table 5 and Figure 3.

### 3.6. Evaluation of Wound Exudate and Edema in Two Groups

The scores of wound exudate and edema in the two groups improved significantly after operation, and gradually improved with the increase of time. The scores of wound exudate and edema in the study group were significantly lower than those in the control group between 3 days and 14 days after operation, and the difference was statistically significant (*P* < 0.05), as manifested in Table 6 and Figure 4.

### 3.7. Evaluation of Inflammatory Factors in the Two Groups

There was no significant difference in TNF-*α* and IL-6 between the two groups on the 1st day after operation (*P* > 0.05). The TNF-*α* and IL-6 in the two groups alleviated significantly with the increase of time between the 3rd and 14th days after operation, and the TNF-*α* and IL-6 in the study group were significantly lower than those in the control group (*P* < 0.05), as manifested in Table 7 and Figure 5.

### 3.8. Safety Evaluation of the Two Groups

The incidence of postoperative complications in the research group was 6.67%, significantly lower than that in the control group (*P* <13.79%), and the difference was statistically significant (*P* < 0.05), as indicated in Table 8 and Figure 6.

## 4. Discussion

Anal fistula is one of the most common diseases in young adults. Anal fistula cannot heal itself without treatment and will recur; therefore, radical surgery should be performed promptly [23]. The wound surface after anal fistula surgery is usually open which makes it susceptible to bacterial attack from feces and intestinal bacteria. This prolongs the wound healing time, which is compounded by abundant perianal nerve endings which makes the postoperative pain intense. Therefore, the wound healing after anal fistula surgery can affect the prognosis of patients [24]. Similar to other surgical wounds, wound healing after anal fistula surgery can be divided into 3 stages, i.e., inflammatory exudate, fibrous tissue hyperplasia, and scar formation [25]. Targeted intervention can effectively relieve postoperative pain, accelerate the disappearance of symptoms, relieve the pain of patients, and promote rapid wound healing.

The results of this study indicated that the postoperative wound exudate, edema score, wound granulation growth score, and VAS score of the two groups improved significantly. In the research group, all these parameters improved gradually with an increase in time. It is suggested that the combination of traditional Chinese medicine fumigation can significantly reduce postoperative pain, reduce wound area, and accelerate wound healing for patients with anal fistula treated with pure red ointment. However, the intervention of postoperative pain in foreign countries is usually based on opioid drugs or local anesthesia, and there is no relevant research on red oil ointment. Linares-Gil et al. [26] highlighted that local preparations of lidocaine plus diclofenac manifested better analgesic efficacy than lidocaine in benign anorectal surgery. The results of the Van et al. [27] study indicated that preoperative analgesia is safe and can reduce pain in the early postoperative period after anorectal surgery. However, the significant amelioration of wound healing after anal fistula surgery in this study may be due to poor meridians, stagnation of qi and blood stasis, and endless carrion after anal fistula surgery.

Red Ointment is a topical preparation developed on the basis of traditional ancient prescriptions which have the effects of clearing away heat and detoxification, collecting dampness and reducing sores, reducing swelling and pain, and growing muscles, thus providing good intervention for patients. This study uses Qingre Zhitong Decoction to implement a combined treatment protocol. A treatment regime that utilises fumigation and washing improves blood circulation on the wound. The warming effect of fumigation and washing can accelerate the blood and lymph circulation on the wound and relieve postoperative pain and edema. At the same time, fumigation and bathing have the effect of secondary cleaning, which can reduce the accumulation of bacteria in the wound and reduce the risk of infection [6, 28, 29]. In the prescription used in this study, *Sophora flavescens* clear away heat and dampness; raw rhubarb releases heat and clear fu organs, remove blood stasis and stop bleeding; *Phellodendron amurense* detoxify, purge fire, and dry heat. The combination of the three above drugs can clear away heat and dampness, reduce swelling and pain, and astringe and produce muscle. The combination of traditional Chinese medicine fumigation and sitz bath combined with red ointment resulted in a more significant curative effect for the patients in the study group.

The results of this study showed that TNF-*α* and IL-6 alleviated significantly with time between 3 days and 14 days after surgery, and TNF-*α* and IL-6 in the study group were significantly lower than those in the control group, and the incidence rate of postoperative complications in the study group was 6.67% significantly lower than that in the control group, suggesting that the combination of red ointment and traditional Chinese medicine fumigation bath can reduce the inflammatory reaction and reduce the possibility of postoperative complications after anal fistula surgery. Qu et al. [30] found 375 chemical components in the 5 main herbal medicines in the prescription of traditional Chinese medicine fumigants for healing. Of the 375 chemical constituents, 59 are active compounds. In addition, 325 target genes of 16 active compounds were obtained in 3 herbs. Functional enrichment analysis established that these overlapping genes were significantly associated with immune response, antibiotic biosynthesis, and complement and coagulation cascades. An integrated network of 133 nodes (8 disease nodes, 3 drug nodes, 8 components, 103 target gene nodes, 7 GO nodes, and 4 pathway nodes) was constructed.

In another study by Qu et al. [31], it was publicized that the healing-promoting fumigation prescription is an effective herbal fumigant, and HE staining demonstrated that CYXX treatment reduced the infiltration of inflammatory cells. A total of 472 DEGs were identified, including 141 upregulated genes and 331 downregulated genes. These genes were significantly associated with skin development, xenobiological stimulation, and inflammation; the concordance rate of RT-qPCR and sequencing results were 83.33%, displaying the high relative reliability of sequencing results. These results are consistent with those of this study, all of which confirm the effectiveness of the combination of traditional Chinese medicine fumigating, washing, sitz-bath, and red ointment in the treatment of postoperative patients with anal fistula.

The effect on the research group level of inflammation is more significant, probably because red ointment is composed of red liters, alum, realgar, and cinnabar. Alum has broad-spectrum antibacterial effect leading to the death of bacteria; realgar has an inhibitory effect on the growth of various dermatophytes; and lead pills can kill bacteria and inhibit mucus secretion [32]. In the fumigated sitz-bath formula, studies have also confirmed that the flavonoids and alkaloids of *Sophora flavescens* can inhibit a variety of bacteria, fungi, etc. [33]. Rhubarb has anti-infection and ameliorate human immunity, and Phellodendron extract has been proved to inhibit bacterial growth, inhibit the expression of body inflammatory factors, and accelerate wound healing through TGF-*β*1 [34].

This study, however, had its limitations such as the small sample size used as the study population. The small sample size makes the accuracy of these results difficult to validate. The other limitation of this study was the short postoperative observation duration which implies that long-term effects are not accounted for in this study. As recommendations for future studies, the researcher proposes an increase in study population size as well as extending the postoperative observation period. Additionally, the authors propose the use of these research findings as a baseline for further studies with the intention of developing standard protocols for using this therapy.

## 5. Conclusion

To sum up, the intervention of traditional Chinese medicine fumigation and sitz-bath combined with red ointment for anal fistula patients after operation can effectively reduce wound healing time, ameliorate postoperative pain, and reduce inflammation levels. These findings can be used to develop guidelines and standard protocols that can be followed by anal fistula patients postoperatively to manage wound healing at their homes.

## Figures and Tables

**Figure 1:** Comparison of pain scores between the two study groups.

**Figure 2:** Comparison of wound healing time between two groups (compared with the control group,^*∗*^*P* < 0.05).

**Figure 3:** Comparison of the growth of granulation in wounds between two groups (compared with the control group, ^*∗*^*P* < 0.05, compared with the 7th day, #*P* < 0.05).

**Figure 4:** Evaluation of wound exudate and edema between the two groups on different days (compared with the control group, ^*∗*^*P* < 0.05, compared with the 7th day, #*P* < 0.05).

**Figure 5:** Evaluation of inflammatory factors in two groups (compared with the control group, ^*∗*^*P* < 0.05, compared with the 7th day, #*P* < 0.05).

**Figure 6:** Incidence of postoperative complications in the two groups.

**Table 1:** Baseline information comparison between groups.

Information		Control group (*n* = 58)	Research group (*n* = 60)	*P* value
Gender (*n*, %)	Male	35 (60.34)	37 (61.67)	6
	Female	23 (39.66)	23 (38.33)	0.681
Age, mean SD, years		40.51 ± 9.14	42.73 ± 8.54	0.224
Disease duration, mean SD, years		1.25 ± 1.33	1.26 ± 1.03	0.824

**Table 2:** Evaluation of the efficacy between two groups.

Group	Research group (*n* = 60)	Control group (*n* = 58)	X2 Index	P Index
Heal	28	20		
Effective	16	18		
Slight	14	16		
Ineffective	2	4		
Total efficiency	58 (96.67%)	54 (93.10%)	12.534	0.001

**Table 3:** Comparison of pain scores between the two groups.

Group	Research group (*n* = 60)	Control group (*n* = 58)	t Index	P Index
Postoperative 3d	3.26 ± 0.75	3.97 ± 0.54	5.453	0.007
Postoperative 7d	1.84 ± 0.14	2.37 ± 0.65	6.746	0.003
Postoperative 14d	0.92 ± 0.21	1.13 ± 0.34	7.534	0.001

**Table 4:** Comparison of wound healing time between the two groups.

Group	Research group (*n* = 60)	Control group (*n* = 58)	t Index	P Index
Healing time (d)	21.15 ± 3.22	25.41 ± 5.28	10.534	0.001

**Table 5:** Comparison of the growth of granulation in wounds between the two groups.

Group	Research group (*n* = 60)	Control group (*n* = 58)	t Index	P Index
Postoperative 3d	0.35 ± 0.05	0.61 ± 0.11	10.534	0.002
Postoperative 7d	0.16 ± 0.05	0.39 ± 0.12	11.415	0.001
Postoperative 14d	0.02 ± 0.01	0.23 ± 0.04	11.962	0.001

**Table 6:** Evaluation of wound exudate and edema in the two groups.

Group		Research group (*n* = 60)	Control group (*n* = 58)	t Index	P Index

Wound exudate score	Postoperative 3d	1.54 ± 0.31	1.98 ± 0.25	8.416	0.003
	Postoperative 7d	0.85 ± 0.22	1.12 ± 0.29	9.534	0.002
	Postoperative 14d	0.42 ± 0.06	0.84 ± 0.12	12.318	0.001

Wound edema score	Postoperative 3d	1.46 ± 0.21	2.35 ± 0.25	10.543	0.001
	Postoperative 7d	1.05 ± 0.11	1.54 ± 0.29	11.417	0.001
	Postoperative 14d	0.16 ± 0.03	0.29 ± 0.08	12.537	0.001

**Table 7:** Evaluation of inflammatory factors in two groups.

Group		Research group (*n* = 60)	Control group (*n* = 58)	t Index	P Index

TNF-*α* (mg/L)	Postoperative 3d	20.15 ± 3.42	21.23 ± 4.55	0.845	0.716
	Postoperative 7d	15.26 ± 2.54	19.35 ± 3.68	8.456	0.017
	Postoperative 14d	11.42 ± 2.51	13.26 ± 3.17	10.234	0.001

IL-(ng/L)	Postoperative 3d	15.28 ± 3.08	14.29 ± 5.32	0.146	0.872
	Postoperative 7d	10.62 ± 2.23	12.19 ± 4.16	9.463	0.007
	Postoperative 14d	7.65 ± 1.17	10.58 ± 2.15	12.374	0.001

**Table 8:** Safety evaluation of two groups.

Group	Research group (*n* = 60)	Control group (*n* = 58)	X2 Index	P Index
Wound bleeding	1	3		
Urinary retention	0	2		
Rash	0	2		
Wound infection	1	1		
Total incidence	2 (6.67%)	8 (13.79%)	9.534	0.012

## Data Availability

The data used to support the findings of this study are available from the corresponding author upon request.
